# The Role of Health Education in Vaccination Nursing

This article has been retracted.

**DOI:** 10.1155/2022/6078846

**Published:** 2022-04-18

**Authors:** Mengjiao Yao, Xiaoping Gu, Yujie Mo, Chunjing Xia, Liwei Tang

**Affiliations:** Jiangqiao Community Healthcare Center, Jiading, Shanghai, China

## Abstract

The role of health education in vaccination is very important. Through various forms of activities, comprehensive and systematic education of health knowledge for people can promote students and others to be aware of vaccination and actively cooperate with vaccination work. Therefore, this article intends to conduct an in-depth study of the role of health education in prevention and treatment and to enhance people's awareness of vaccination. This article mainly uses questionnaire survey method, interview method, and controlled experiment to explain and analyze the effect of health education. The subjects of this questionnaire are students, parents, and staff. They have mixed reviews for its role in vaccination, but the overall situation is positive. 239 out of 500 people believe that health education can reduce allergic reactions and improve the effectiveness of vaccines. In the control experiment, after health education and publicity training, the parents of the observation group were significantly better than the control group in terms of mastering the relevant knowledge of vaccination, successfully vaccinating unplanned vaccines, etc. This shows that the importance of health education in vaccination care is incomparable.

## 1. Introduction

Our country's disease prevention work mainly focuses on public health. Factors such as large population, poor sanitation, and unbalanced economic development have affected people's understanding of disease knowledge. Health education is a kind of knowledge dissemination that focuses on prevention and combines prevention and treatment. It achieves the purpose of improving people's ideological awareness and enhancing the role of vaccines by cultivating and educating people in a certain degree of comprehensive physical and psychological qualities.

There are countless research results on the role of health education in vaccination care. For example, Wang et al. emphasized that in view of the problems existing in mass vaccination in schools, if targeted preventive care measures can be taken, the quality of medical care and the safety of vaccination can be greatly improved [1]. Tang pointed out that the scientific development of vaccination nursing work has a good effect on relieving the nervousness of children during vaccination, thereby promoting the success rate and safety of vaccination [2]. Yang and Wu explored the role of parental health education and nursing intervention in reducing the side effects of DPT vaccination among high school students. Parental health education and care intervention can significantly improve the understanding of the DPT vaccine among the parents of students who have received the DPT vaccine, thereby significantly reducing the awareness rate of the DPT vaccine [3]. Therefore, this article also follows the research line of other scholars and conducts in-depth exploration of the role of health education in vaccination care.

This article first studies the relevant theories and knowledge of health education. Then, a brief description of vaccination care is given. Afterwards, the function and performance of the design of the vaccination information management system were analyzed. Finally, through questionnaire surveys and experiments, an in-depth study of the role of health education in vaccination care was carried out, and data results were obtained [4]. The data show that through scientific health education, parents' cognition, the reduction of children's anxiety, and the success rate of vaccination can be significantly improved. The experiment proved the necessity of health education.

## 2. The Role of Health Education in Vaccination Care

### 2.1. Health Education

Health education is a scientific education that focuses on prevention and combines treatment. Its purpose is to let the audience have a correct and comprehensive understanding of the disease, improve people's self-protection ability, and enable them to receive effective care in social life. Health education is through the comprehensive and systematic shaping of people's physical and psychological factors so that they can establish a correct, positive, and self-improving ideology. The role of health education in vaccination care is very important [5, 6].

Health education is a systematic project, which requires systematic and planned planning as well as continuity. In terms of health knowledge, it mainly starts from the two perspectives of life care and social hygiene. As people's understanding of diseases continues to deepen, more and more knowledge about vaccination and nursing knowledge, methods, and approaches have begun to spread. The so-called health is a comprehensive good state of physique, psychological quality, and personality quality that combines a good mental state with a good physical shape [7, 8].

Health education can effectively improve people's misunderstanding of diseases, lifestyles, and behaviors, so as to achieve the purpose of vaccination and nursing. In health promotion and education, we must fully consider the individual differences of each patient, family environment, and other factors. Let more people in the whole society understand diabetes knowledge and prevention methods through publicity boards and playing video clips. Regularly organize “sports and fitness” activities to enable the general public to correctly understand the importance and role of sports in improving physical fitness. Actively cooperate with community neighborhood committees or residents' committees to conduct physical examinations for people with diabetes and guide them on how to vaccinate [9, 10].

In daily work, the importance of health education should be strengthened, and comprehensive and systematic publicity should be organized regularly to enable people to fully understand how to properly use and wear disease prevention equipment and related knowledge. At the same time, it can be spread through platforms such as WeChat official account.

Effective antibodies can be produced after vaccination, and such diseases will not occur after future contact, and vaccination is now free [11, 12].

Pay attention to the health education of parents. Parents should observe closely and do not give children antibiotics without authorization [13, 14].

Medical staff should pay attention to giving different nursing care to students' psychological reactions in different periods [15, 16].

### 2.2. Vaccination Care

Vaccination care refers to regular education of healthy patients so that they understand the disease and how to treat it and cultivate good habits in daily life. Through regular physical examinations, problems are found and solved in time.

Health education plays a very important role in vaccination care. It can help people understand their physical health and take corresponding measures to effectively control diseases. Nurses have a comprehensive knowledge and understanding of health education. In the actual nursing process, implement it to every construction worker, and all participants are required to strictly abide by the relevant regulations and take corresponding measures for different situations.

Regular lectures on vaccination and nursing knowledge: let parents and family members understand what problems need to be paid attention to in daily work and how to better and timely solve the various new situations in the medical history, discover potential risk factors, and control the development trend of the disease.

In health education, we can improve the staff's awareness of disease knowledge and awareness of disease prevention through professional training and qualification examinations. At the same time, it is necessary to strengthen communication with patients and their families.

Strengthen health education and publicity to train people through lectures, playing DVDs, etc., so that everyone can understand the importance of vaccination care and strengthen the relationship between people's disease and vaccination work. At the same time, some simple and easy-to-operate activities should be carried out in the hospital to increase the public's awareness of participation. Organize a regular theme activity with the theme of “Prevention and Treatment of Diseases” and distribute corresponding materials.

### 2.3. Design of Vaccination Information Management System

#### 2.3.1. Data Mining Technology in the Management System

In the information management of vaccination, special technology is needed to sort and analyze the information and data. Based on the dimensionality of the data involved in the rule, association rules can be divided into single-dimensional and multidimensional. Its definition can be expressed as follows:

(1) $$\begin{array}{c} \text{Support}\left(P\Rightarrow Q\right)=P\left(P\cup Q\right),\\ \text{Confidence}\left(P\Rightarrow Q\right)=F\left(P|Q\right). \end{array}$$

Among them, the degree of support for association rules *P*⇒*Q* is *F*(*P* ∪ *Q*). These data analysis techniques can be directly applied to the vaccination information data warehouse.

#### 2.3.2. Vaccination Management

Vaccination is a welfare policy of the state to ensure the healthy growth of children and avoid contracting diseases. Vaccination information will be entered into the file as a required document for future enrollment. The production, packaging, and distribution of vaccines are also strictly controlled by the relevant departments, and the distribution is agreed.

In order to ensure the accuracy of each link in the vaccination process for children, each link will confirm the information and enter it into the computer, and the vaccine information will also be archived.

As for which vaccines to be vaccinated at different time periods, publicity brochures will also be formulated in advance and distributed to parents, which will also clearly indicate the adverse reactions of some vaccines.

The entire vaccination process plays a vital role in improving children's physical health and reducing the infection rate of group diseases and high-incidence diseases.

## 3. Experimental Investigation

### 3.1. Survey Object

This article first interviewed the vaccinated staff of the health center, mainly to explore the attitude and knowledge of the practitioners about the job. There is a total of 80 staff members under investigation. This article designs a relevant questionnaire to conduct a questionnaire survey on them.

Then, select 100 students who need vaccinations as the observation group. Among them, 52 were boys and 48 were girls. The vaccinated students are in good health and normal development. There is no special sensitivity reaction to vaccination. In addition, 90 students who need to receive vaccination were selected as the control group, of which 54 were boys and 46 were girls. There is no significant difference in gender between the two groups of experimental students, and they are comparable.

In addition, this article also invited the parents of the students to conduct surveys and interviews. Among the guardians of the survey subjects, there are up to 120 student mothers, 80 student fathers, and 30 grandparents.

### 3.2. Health Education Methods

Health education is a step that we all need to focus on throughout the vaccination process. Health education is not only a unilateral propaganda by medical staff but a mode of passive acceptance by parents. This mode can easily lead to parents' irritability and poor results.

Healthcare workers should consider innovative formats, such as educational video clips that encourage parents and children to watch together. In addition, you can also consider printing some storybooks and picture books to promote health education knowledge in the stories. Of course, giving children some small toys printed with health education can also have a good publicity effect.

Of course, the above method will inevitably incur costs, so the relevant part needs to issue funds to the community service station. Through the above methods, children can not only realize the harm of disease and can actively stay away from the source of disease in their daily life but also can enhance parents' awareness of vaccination.

### 3.3. Questionnaire Survey Method

The survey objects of this paper are parents and the staff of the community service station. The survey site is the community service station. The survey time is selected as weekends, because weekends are the peak time for parents to bring their children to vaccinate. In the form of face-to-face paper questionnaires, parents' real views on vaccination and health education, as well as their satisfaction with the vaccination process, were obtained.

In addition, we also distributed paper questionnaires to the staff of 10 community service workstations, mainly to investigate the difficulties they face during the usual vaccination process so as to propose solutions.

## 4. Analysis of Survey Results

### 4.1. Main Difficulties Faced by Vaccination

First of all, this article intends to analyze the main difficulties faced by vaccination. According to the survey data of the staff, we can see that 64 of the 90 staff are concerned about the 5 aspects of vaccination, namely, insufficient assistance, negative reports, noncooperation of the masses, weak team, and lack of salary and labor. There are great opinions on matches, etc. The specific data are shown in Table 1.

As shown in Figure 1, we can judge that the staff attach great importance to the problem of vaccination, and they believe that the two aspects of insufficient aid and the impact of negative reports have a negative impact on the work. This is enough to show that the health education work for vaccination is not yet in place, and the country's management is not perfect. Among them, only 14 people disagreed with these issues, and 12 others did not comment on it.

### 4.2. Parents' Satisfaction with the Work of Vaccination Clinic

Secondly, this article invites parents to conduct a questionnaire survey and found that the degree of satisfaction with the overall outpatient clinic, the number of consultations, waiting for observation, postevent precautions, sanitary conditions, and service procedures are also different. On average, about 160 people are satisfied with these 6 places, and about 42 people are dissatisfied with these places. The details are shown in Table 2:

As shown in Figure 2, we can clearly see that the parents are most satisfied with the sanitary condition of the vaccinated health center, and then they are satisfied with the service process. The most unsatisfactory thing is the number of visits in the outpatient department. As people are now more and more aware of the importance of vaccination, they attach great importance to vaccination. However, there is a time limit for vaccination, and there are not many consultations, so parents feel distressed about this.

### 4.3. Comparison of Effects between the Observation Group and the Control Group

Then, this article needs to understand the grouping situation. After conducting health education and publicity training for parents, 97 of the 100 parents of students in the observation group have knowledge of vaccination. 94 cases were successfully vaccinated with unscheduled vaccines, and 95 cases were qualified. Among the 100 parents of students in the control group, 61 parents successfully mastered vaccination-related knowledge. 68 students were successfully vaccinated with unscheduled vaccines, and 72 students passed the vaccine. According to the data comparison, it can be clearly seen that the inoculation effect of the observation group is better than that of the control group. The details are shown in Table 3.

As shown in Figure 3, we can find that the vaccine qualification rate, unplanned qualification rate, and knowledge mastery rate of the observation group and the control group are better than those of the control group. In terms of vaccine qualification rate, the observation group is 27% larger, and in the unplanned qualification rate, the observation group is 22% larger. In terms of knowledge, the observation group can reach 97%. This shows that health education plays a great role in vaccination and can have an impact on the effectiveness of vaccines.

### 4.4. The Role of Health Education in Vaccination

Finally, this article conducts research on reducing adverse vaccine reactions, increasing satisfaction, improving vaccine effects, and reducing the occurrence of allergic reactions from the three perspectives of students, parents, and medical staff. From the data collection, it can be found that 142 people think that health education can reduce the occurrence of allergic reactions, 96 people think it can improve the effectiveness of the vaccine, and 153 people say it can increase satisfaction. Another 122 people said that health education would reduce the adverse effects of the vaccine. The details are shown in Table 4.

As shown in Figure 4, we can see that in the student population, most of them believe that health education can reduce the occurrence of allergic reactions. The proportion is 36.8%. In the parent group, most of them think that health education can improve their satisfaction and increase their awareness of vaccination. The proportion is 39.1%. In the staff group, they believe that health education can improve the effect of vaccination. The proportion is 35%.

## 5. Conclusion

The role of health education in vaccination care is very important. The use of purposeful and comprehensive preventive and healthcare measures and scientific and effective guidance to the public can enable people to develop good living habits and promote physical and mental development. Targeted activities aimed at reducing diseases, enhancing physical and mental harmonious development, and promoting a sustainable and virtuous circle of society. At this stage, the most powerful disease prevention method in our country is vaccination, and many people have great doubts about the effect of this method. Through the experimental research in this paper, it is found that the use of scientific health education has a significant positive impact on infant vaccination care. It can not only effectively improve parents' scientific understanding of vaccine injection but also improve the effect of vaccine injection objectively.

## Figures and Tables

**Figure 1:** Major difficulties faced in vaccination efforts.

**Figure 2:** Parents' satisfaction with the vaccination clinic work.

**Figure 3:** Effect comparison between the observed and control groups.

**Figure 4:** The role of health education in vaccination.

**Table 1:** Major difficulties faced in vaccination efforts.

	Agree	Disagree	General
Insufficient superior subsidies	18	4	1
Negative reports impact	19	2	1
The masses do not cooperate	13	3	2
Weak personnel team	6	2	3
Revenue is not linked to the workload	8	3	5

**Table 2:** Parents' satisfaction with the vaccination clinic work.

	Satisfied	Unsatisfied	General
General outpatient service	161	42	31
Number of opening visits	119	68	39
Waiting for planting to stay	142	61	32
Matters needing attention afterwards	163	36	26
Sanitary conditions	192	22	17
Service process	183	20	22

**Table 3:** Effect comparison between the observed and control groups.

	Observation group	Control group
Number	100	100
Vaccine pass rate	95	68
Out planned qualified rate	94	72
Knowledge mastery rate	97	61

**Table 4:** The role of health education in vaccination.

	Students	Parents	Workers
Reduce adverse vaccine reactions	42	40	40
Increase satisfaction	51	92	10
Improve vaccine effect	30	39	27
Reduce the occurrence of allergic reactions	69	51	22

## Data Availability

The data used to support the findings of this study are available from the corresponding author upon request.
